# Correlation between Imaging Features and Pathological Stages of Primary Lung Tumors Based on Nanocontrast Agents

**DOI:** 10.1155/2021/2343299

**Published:** 2021-11-08

**Authors:** Jin Li, Qian Xu, Cunhua Mao, Yuliang Liu

**Affiliations:** ^1^Department of Radiology, Jinan Third People's Hospital, Jinan, Shandong, China; ^2^Department of Image, Jinan Municipal Hospital of Traditional Chinese Medicine, Jinan, Shandong, China; ^3^Department of Radiology, The Affiliated Hospital of Shandong University of Traditional Chinese Medicine, Jinan, Shandong, China

## Abstract

As one of the conventional methods of lung cancer detection, computed tomography (CT) usually requires the use of contrast agents to enhance the imaging effect. Conventional iodine contrast agents have poor signal-to-noise ratio and are prone to adverse reactions. It is necessary to find more effective and safe contrast agents for CT scans. The gold nanoparticles with secondary electron effect and photoelectric absorption effect can prolong the display time of the patient's blood circulation after being injected into the patient's body, which makes the nanocontrast agent a research hotspot in the field of CT imaging. In this study, ultrasmall gold nanoclusters with a diameter of about 5 nm were used as the contrast agent in CT scans. It was found that CT scans based on nanocontrast agents can obtain high-quality lung cancer imaging images, and the patient has no obvious adverse reactions. When observing the CT image, it was found that the stage of lung cancer patients can be clearly distinguished through the CT scan image. When analyzing the consistency of CT imaging and pathological classification, the Kappa value was 0.810, indicating that the two have a high degree of consistency. Therefore, this study believes that the imaging characteristics of primary lung tumors based on nanocontrast agents are highly correlated with their pathological types.

## 1. Introduction

Lung cancer is a malignant tumor that poses a great threat to human life and health. Its morbidity and mortality rate ranks first among malignant tumors in the world, and the morbidity and mortality rates are still on the rise [1]. According to relevant epidemiological survey data, the incidence of lung cancer is about 5 : 1 between men and women, among which middle-aged and elderly men are the high-risk population of lung cancer [2]. The specific pathogenesis of lung cancer has not yet been fully understood, but the risk factors that induce lung cancer have gradually become clear. A number of studies have shown that factors such as air pollution, smoking, diet, occupational carcinogens, and genetics can increase the risk of lung cancer [3–5]. This may be the main reason why the incidence of lung cancer has increased year by year as air pollution has increased and the number of smokers has increased. In the early stages of lung cancer, patients often experience symptoms such as irritating cough, increased sputum volume, and loss of appetite [6]. As the disease progresses, symptoms such as blood in the sputum or hemoptysis, chest tightness, chest pain, fever, or difficulty breathing will appear. Without timely and effective treatment, when cancer cells invade the pleura, ribs, and shoulders, the patient's cough and pain symptoms will aggravate and even lead to superior wall vein occlusion syndrome, Horner syndrome, brachial plexus nerve compression, etc. complications [7, 8]. In addition, it may also cause cancer cells to metastasize to the liver, kidneys, and bones, causing systemic malignancy and directly endangering the lives of patients.

At present, there are many treatment methods for lung cancer, and the specific treatment plan should be formulated according to the patient's physical fitness, tumor pathological type, and degree of invasion. Among them, chemotherapy is the most common treatment for lung cancer. Chemotherapy can effectively reduce the growth rate of cancer cells in patients and reduce their spread. However, the chemotherapy cycle is longer, and it will bring obvious complications to the patient, which has a serious impact on the quality of life of the patient. At the same time, as the disease progresses, the difficulty of treatment increases, and the possibility of cure also decreases. Therefore, the early diagnosis of lung cancer through imaging examination and pathological analysis has a positive effect on the treatment and prognosis of patients. X-ray computed tomography (CT) is a technique that uses the different absorption degrees of X-rays by body tissues to image and has been proven to have good imaging effects on solid tissues [9]. However, CT has poor imaging capabilities for blood vessels and usually requires a combination of contrast agents to improve its scanning sensitivity. Due to individual differences, some patients will have adverse reactions to contrast media, which makes the safety of CT contrast media the focus of attention of doctors and patients. With the rapid development of bionanotechnology, CT contrast agents based on nanoprobes have appeared in people's field of vision [10]. Nanoparticles are small in size and can match biomolecules, so they can be made into contrast agents to detect pathological changes in the body. This makes the nanocontrast agent become a research hotspot in CT imaging diagnostic technology. This study is based on the analysis of the correlation between the imaging characteristics of primary lung tumors and different pathological stages based on nanocontrast agents, in order to provide references for the early diagnosis and clinical treatment of lung cancer.

## 2. Materials and Methods

### 2.1. Research Process

Formulate inclusion and exclusion criteria and screen research subjects based on the criteria. Patients who meet the enrollment conditions will be diagnosed by CT scanning before surgery (using nano-CT contrast agent for CT scanning), and pathological diagnosis will be performed after surgery, and the consistency of CT diagnosis and pathological diagnosis will be analyzed (the specific research process is shown in Figure 1).

### 2.2. Research Object

A total of 92 patients with primary lung cancer admitted to our hospital from January 2020 to January 2021 were selected as the research objects. Enrolled patients need to meet the following five inclusion criteria: (1) meet the diagnostic criteria for primary lung cancer [11], (2) all ages > 18 years, (3) volunteer to participate after learning about this study, (4) the mental state is normal and can cooperate to complete the whole study, and (5) no blood system disease. Exclude patients who meet the following conditions: (1) unconsciousness; (2) with severe heart, liver, and kidney insufficiency; and (3) with hypertension, diabetes, and hyperlipidemia.

### 2.3. CT Imaging Instrument and Detection Method

Use Siemens Somatom Definition dual-source CT scanner for image acquisition. Before the scan, inform the patient of the precautions for breathing and holding his breath, and perform a horizontal CT scan of the whole lung during the formal scan. Set the layer thickness (8 mm), voltage (120 kV), current (110 mAs), detector width (32 × 0.6 mm), and pitch (1.0) of the single-source scanning. The dual-source scan mode is used for enhanced scanning, setting the voltage (A tube: 140 kV; B tube: 100 kV), current (A tube: 180 mAs; B tube: 160 mAs), detector width (A after scanning parameters such as 32 × 0.6 mm), slice thickness (1.5 mm), and reconstruction interval (1.0 mm) for both tube and B tube; the two tubes A and B are scanned at the same time to obtain image information. The nanocontrast agent was injected through the cubital vein with a high-pressure injection at a flow rate of 3.0 mL/s. After the nanocontrast agent was injected, 30 mL of physiological saline was injected into the tube at the same flow rate. The CT scan was triggered by the contrast agent bolus tracking software (the arterial phase trigger threshold was 100 HU). The artery was injected with the nanocontrast agent 25 s after the injection, and the vein was injected 30 s after the injection.

### 2.4. CT Scan Standard and Imaging Analysis of Lung

The acquired CT scan images are evaluated by two radiologists with senior professional titles, and a unified determination will be given after discussion when there is a disagreement. The content of the assessment mainly includes the location, shape, edge, density, and boundary of the lesion, and the Tumor-Node-Metastasis (TNM) staging of the patient is clarified according to the imaging characteristics.

### 2.5. Pathological Staging of Primary Lung Tumor

The postoperative lesion tissue of the patient was collected, fixed with 4% formaldehyde, dehydrated with gradient alcohol, embedded in paraffin, and prepared for conventional HE staining (immunohistochemical staining was performed for sections that were still difficult to be diagnosed by conventional HE staining). The diagnosis of pathological staging is jointly agreed by 2 pathologists with senior professional titles.

### 2.6. Consistency Check

Kappa consistency test was used to analyze the consistency of CT scan imaging and pathological detection. The sum of observations in the diagonal unit (Po) and the sum of the expected values in the diagonal unit (Pe) are important indicators in Kappa detection. When Kappa > 0.75, it indicates a high degree of consistency, and Kappa is between 0.40 and 0.75; it indicates a good consistency; Kappa < 0.40 indicates poor agreement. The calculation formula of Kappa consistency test is shown in formula (1).

(1) $$\begin{array}{c} \text{Kappa}=\left(\text{Po}-\text{Pe}\right)÷\left(1-\text{Pe}\right). \end{array}$$

### 2.7. Statistical Analysis

This study used the SPSS v.23.0 and GraphPad Prism v.8.0 software for data analysis. Quantitative data are expressed in the form of mean ± standard deviation. Two-group comparisons and multigroup comparisons were performed by *t*-test and analysis of variance, respectively. The qualitative data is expressed in the form of *n* (%), and the chi-square test is performed. The consistency of the preoperative CT diagnosis staging and postoperative pathological staging was performed by Kappa test. The comparison between all data is *P* < 0.05 indicating that the difference is statistically significant.

## 3. Results and Discussion

### 3.1. Postoperative Pathological Diagnosis Results of the Patient

After pathological examination of the patient's cancer tissues, it was found that among 92 patients with primary lung cancer, 18, 39, 27, and 8 were in stages I, II, III, and IV, respectively (as shown in Figure 2).

### 3.2. Preoperative CT Image Characteristics of Patients

In this study, an ultrasmall gold nanocluster contrast agent was injected into the patient before the CT scan (the transmission electron microscopy image and particle size distribution of the gold nanocluster are shown in Figures 3(a) and 3(b)) to extend the photography time and enhance the imaging clarity. Under the action of the nanocontrast agent, we can clearly observe the patient's lung imaging characteristics. By analyzing the imaging characteristics of lung cancer patients at different stages, we found that the lungs of patients with lung cancer can see sheet consolidation, ground glass shadows, and burrs, with clear and irregular boundaries. And we can clearly observe that with the aggravation of the patient's disease, the number of enlarged lymph nodes in the mediastinum increased significantly, and the mass in the lower right part of the lung increased significantly. These results suggest that CT imaging based on nanocontrast agents can effectively reflect the staging of lung cancer patients.

### 3.3. Analysis of Consistency between CT and Postoperative Pathological Staging

It can be seen from Table 1 that CT using nanocontrast agents has excellent consistency between the pathological staging diagnosis results of lung cancer patients and the surgical pathological diagnosis results (Kappa = 0.810). And it can be seen from the comparative data (as shown in Figure 4) that the diagnostic coincidence rate of stages III and IV lung cancer using nanocontrast agent CT is higher than that of stages I and II. This may be because the lung tissue of patients with advanced lung cancer is more infiltrated by cancer cells, and the blood vessels in the lungs are obviously damaged. Under the action of the nanocontrast agent, CT can clearly reflect the patient's lung lesions.

### 3.4. Discussion

Lung cancer is a malignant tumor with high morbidity and mortality worldwide. Because of its lack of typical symptoms in its early stage, it causes high misdiagnosis and missed diagnosis [12, 13]. Most patients are already in the advanced stage at the time of diagnosis, which greatly reduces the survival rate of lung cancer patients. Therefore, the early detection and treatment of lung cancer is very important, and how to improve the clinical diagnosis of lung cancer has become a hot spot in clinical research. Pathological examination is the gold standard for diagnosis of lung cancer. It can accurately understand the pathological stage of patients and provide reference for subsequent treatment. However, the pathological examination is an invasive operation and can cause damage to the patient's body. Imaging examinations are widely used in the diagnosis of many diseases due to their noninvasive advantages [14, 15]. At present, the imaging examinations used for the diagnosis of lung cancer mainly include X-ray examination, magnetic resonance (MRI), and CT. X-rays can detect abnormal signs of the lungs at an early stage, but X-rays have many hidden areas for detection and are prone to missed diagnosis [16]. MRI has good resolution and can clearly distinguish the mediastinum, hilar vessels, masses, and lymph nodes, but the lungs are high in air content and are prone to artifacts [17]. Due to its high resolution, CT has the characteristics of fast scanning time and clear images and is not easily affected by lung gas. At the same time, CT can also find hidden areas of X-ray detection [18, 19].

With the continuous development of CT technology, the scope and indications that can be examined have been continuously expanded, which makes CT a routine examination in the imaging department. In the process of clinical CT examination, contrast agents are usually used to improve the display rate of lesions and enhance the integrity of blood perfusion and blood-brain barrier. Iodine contrast agent is a traditional CT contrast agent, which has been proven to enhance the effect of CT imaging. However, studies have shown that some patients experience symptoms of cough, chest tightness, nausea, or fever after using iodine contrast agents and even severe adverse reactions such as convulsions, convulsions, and loss of consciousness [20, 21]. In addition, there may be leakage of iodine contrast agent at the injection site, causing pain, swelling, and necrosis of the subcutaneous tissue. In addition, there are many precautions for the use of iodine contrast agents. For example, when using iodine contrast agents, patients need to use nephrotoxic drugs, mannitol, diuretics, and other drugs for the disease. Wang et al. confirmed in his research that the signal-to-noise ratio of iodine contrast agent is relatively poor, and there are certain biological safety risks [22]. Therefore, finding new and effective CT contrast agents has become the focus of research by many scholars and clinicians.

With the rapid development of nanotechnology in medicine, gold nanoparticles with secondary electron effects and photoelectric absorption effects are used as contrast agents for cancer diagnosis. Injecting gold nanoparticles into the patient's blood can prolong the CT display time of the patient's blood circulation and obtain high-quality medical images [23]. In his research, Lee et al. stated that gold nanoparticles based on heavy atoms can increase the circulation time and enhance the effect of CT imaging [24]. However, some studies have found that when the diameter of the nanoparticles is large, the contrast agent is easy to accumulate in the liver and spleen of the patient, which may cause cytotoxicity [25]. This limits the application of gold nanoparticles in X-ray CT scanning. The ultrasmall gold nanoclusters have a diameter of only about 5 nm, which has strong osmotic metabolism and is easier to be cleared by the body [26–30]. Therefore, ultrasmall gold nanoclusters have become a hot spot material for CT contrast agents due to their easy metabolism, low toxicity, and high uptake properties. In this study, ultrasmall gold nanoclusters were used as the contrast agent for CT detection, and high-quality CT scan images were obtained, and the patient had no obvious adverse reactions. When observing the CT image, it was found that the stage of lung cancer patients can be clearly distinguished through the CT scan image. When analyzing the consistency of CT imaging and pathological classification, the Kappa value was 0.810, indicating that the two have a high degree of consistency. Therefore, this study believes that the imaging characteristics of primary lung tumors based on nanocontrast agents are highly correlated with their pathological types.

## 4. Conclusion

In summary, in this study, ultrasmall gold nanoclusters with a diameter of about 5 nm were used as the contrast agent for CT scanning, and high-quality imaging images were obtained after CT scanning. When the patient's imaging staging results and pathological staging results were analyzed for consistency, it was found that the two had a high degree of consistency. Therefore, this study believes that the imaging characteristics of primary lung tumors based on nanocontrast agents have a high correlation with their pathological types, and the pathological staging of patients can be judged by the imaging characteristics of patients.

## Figures and Tables

**Figure 1:** Research flow chart.

**Figure 2:** Distribution of the number of patients in different stages.

**Figure 3:** Gold nanocluster CT contrast agent: (a) transmission electron micrograph of nanoparticles; (b) diameter distribution diagram of nanoparticles.

**Figure 4:** The coincidence rate of CT diagnosis of lung cancer pathological staging after using nanocontrast agent.

**Table 1:** Comparison of computed tomography diagnosis results and pathological diagnosis results.

CT diagnostic staging	Pathological diagnostic staging				Total
	I	II	III	IV	
I	17	3	2	0	22
II	1	36	5	0	42
III	0	0	20	1	21
IV	0	0	2	7	7
Total	18	39	27	8	92

## Data Availability

All the raw data could be accessed by contact the corresponding author if any qualified researcher need.
